The article "A novel TUBG1 mutation with neurodevelopmental disorder caused by malformations of cortical development" was retracted in 2023. Reasons: suspected computer-generated content; unreliable results or conclusions; concerns about the data; concerns about the results or conclusions.

# A novel *TUBG1* mutation with neurodevelopmental disorder caused by malformations of cortical development

**DOI:** 10.1155/2021/6644274

**Published:** 2021-02-26

**Authors:** Ru Shen, Zhen Zhang, Yu Zhuang, Xiaohong Yang, Lifen Duan

**Affiliations:** ^1^Division of Laboratory, Kunming Children's Hospital affiliated with Kunming Medical University, Kunming 650028, China; ^2^Institute of Pediatrics, The Kunming Children's Hospital, Key Laboratory of Child Critical Disease Research of Yunnan Province, Kunming 650028, China; ^3^Division of Neurology, Kunming Children's Hospital affiliated with Kunming Medical University, Kunming 650028, China

## Abstract

Neurodevelopmental disorder caused by malformations of cortical development is a rare neurological disease. Heterozygous missense variants in the *TUBG1* gene lead to malformations of human cortical development, which further result in intellectual disability, developmental retardation, and epilepsy. To the best of our knowledge, only thirteen patients and a total of nine pathogenic *TUBG1* variants have been described in the published literature. This study reports the case details and genetic data analysis of a girl (aged 8 years, 9 months) with developmental delay, psychomotor regression, epilepsy, and left external ear deformity. A novel *TUBG1* mutation was identified by whole-exome sequencing and Sanger sequencing, confirming that this mutation may be the cause of the neurodevelopmental disorders. This case report characterizes the phenotypic spectrum, molecular genetic findings, and functional consequences of novel pathogenic *TUBG1* variants in neurodevelopmental disorders caused by cortical development malformations.

## 1. Introduction

Neurodevelopmental disorders caused by malformations of cortical development (MCD) are rare diseases with high clinical heterogeneity. The main clinical features of MCD include motor impairment, intellectual disability, early-onset epilepsy, and cortical malformations (including lissencephaly, polymicrogyria, microlissencephaly, pachygyria, and simplified gyration) [1, 2]. There are many reasons for MCD such as KIF5C gene mutation [3]. However, the cortical and extracortical brain phenotypes observed are largely dependent on the specific tubulin gene affected.

Tubulin genes play a key role in several pathways of cortical development. Mutations in these genes may cause specific brain malformations strictly associated with epilepsy [4]. Mutations affecting seven genes encoding alpha- (*TUBA1A*), beta- (*TUBB2A*, *TUBB2B*, *TUBB3*, *TUBB4A*, and *TUBB*), and gamma-tubulin (*TUBG1*) have been identified in individuals with a range of malformations of cortical development (MCDs) [5].

The article "A novel TUBG1 mutation with neurodevelopmental disorder caused by malformations of cortical development" was retracted in 2023. Reasons: suspected computer-generated content; unreliable results or conclusions; concerns about the data; concerns about the results or conclusions.

In mammalian cells, *γ*-tubulin is highly conserved and often encoded by two genes. Humans have *γ*-tubulin 1 and *γ*-tubulin 2 *(TUBG1* and *TUBG2*) [6]. *TUBG1* is thought to be ubiquitously expressed, whereas *TUBG2* expression appears to be restricted to the brain [6, 7]. Mutations in the *TUBG1* gene located on chromosome 17q21 are one of the causes of neurodevelopmental disorders caused by MCD [8, 9]. *TUBG1* encodes *γ*-tubulin, which is highly expressed in the developing fetal brain as a component of centrosomes [8].

*TUBG1* plays an integral role in microtubule nucleation, thereby affecting microtubule-dependent mitosis and brain development [10–12]. Poirier et al. introduced variants in the *γ*-tubulin gene that interfered with microtubule nucleation in *Saccharomyces cerevisiae*. The suppression of *TUBG1* in mice in utero also arrested neuronal migration [13]. Ivanova et al. studied seven MCD-related identified variants in *TUBG1*, and the study results suggest that disease-related *TUBG1* variants exert their pathogenicity by affecting microtubule dynamics rather than centrosomal positioning or nucleation ability [5].

*TUBG1* mutations in neurodevelopmental disorders caused by MCD exhibit a relatively limited mutational spectrum [14]. Only nine pathogenic variants in thirteen cases of *TUBG1* mutations have been reported, and the main phenotypes are epilepsy combined with retardation of intelligence, language, and motor development. In this article, we describe a novel pathogenic variant of the *TUBG1* gene (c.751A>T p.N251Y) identified through whole-exome sequencing (WES) in a Chinese patient who presented epilepsy, intellectual disability, speech impairment, and left external ear deformity; these findings may serve to improve diagnosis, management, and research on neurodevelopmental disorders caused by MCD.

## 2. Materials and Methods

### 2.1. General Patient Information and Ethical Considerations

This study was reviewed by the Medical Ethics Committee of Kunming Children's Hospital affiliated with Kunming Medical University. Informed consent for genetic analysis was obtained from the parent. Clinical information and blood specimens were obtained from the patient and her family members.

The patient was a girl who was 8.75 years old and was the second child born to nonconsanguineous parents. She had a height of 1.17 meters, a weight of 18 kg, short stature, left auricle deformity, and pectus excavatum (Figure 1), and she had been diagnosed with epilepsy for 7 years. The patient experienced a relapse of epilepsy and came to the neurology outpatient department of our hospital. The parent complained that there was no obvious cause of the afebrile convulsions 5 times a day during the awake period when the child was 1 year old. The condition manifested as a sudden turning of the eyes, no response to calling, and limb twitching, (but no foaming at the mouth, or incontinence). Each episode lasted 10-20 minutes followed by relief, lethargy, and normal mental activity after wakening. The patient was diagnosed with epilepsy in other hospitals and was administered herbal medicine for more than 3 years to control seizures.

The article "A novel TUBG1 mutation with neurodevelopmental disorder caused by malformations of cortical development" was retracted in 2023. Reasons: suspected computer-generated content; unreliable results or conclusions; concerns about the data; concerns about the results or conclusions.

The patient had an attack every half month to a month while receiving medication. She was then treated with sodium valproate, topiramate, and levetiracetam. The drug dosage was unknown at that time. After taking the medicines for 3 years, she stopped taking it because of poor eating during the course of the treatment, and the seizures recurred after stopping the medicines.

The patient underwent thorough examination, including physical growth examination, laboratory examination, imaging examination, and behavior development assessment. Although the patient was 8.75 years old, her cognitive abilities were equivalent to those of a child aged 2-3 years. She was hyperactive and could not count or perform calculations. She could repeat adult language, but she could not communicate with others and could not eat alone or care for herself. She fell easily when walking fast. She was admitted to the neurology department of our hospital due to epilepsy and mental retardation.

### 2.2. Imaging Examination

The patient's conventional 12-lead electrocardiogram showed sinus arrhythmia and some T wave changes.

The patient's electroencephalogram (EEG) on August 16, 2019 showed that the EEG was abnormal when she was awake. Specifically, the background delta activity increased, and bilateral frontal and occipital sharp waves and sharp slow waves were released. Head CT showed that the white matter area of the bilateral lateral ventricles was reduced and the shape was irregular. CT of the patient's head showed that the white matter area of the bilateral lateral ventricles was reduced and that the shape was irregular.

Head MRI (August 16, 2019) revealed the following (Figure 2): (1) The gyrus of each lobe of the bilateral cerebral hemispheres is thick, the cortex is thickened, the surface is smooth, the sulci are few and shallow, and the bilateral ventricles are enlarged. No abnormal signal foci were found in the parenchyma of the brain. (2) The ventricular system was enlarged and the left temporal extracerebral space was widened. (3) The structure of the cerebellar hemisphere was poor.

### 2.3. Whole-Exome Sequencing and Genome Copy Number Analysis

First, we extracted genomic DNA from the peripheral blood of the proband and her family; NGS-based genetic testing was performed using Agilent SureSelect capture (Agilent, Santa Clara, California) and purified the DNA by amplification. We used the high-throughput sequencing platform (Illumina NovaSeq6000, USA) to detect the exon regions and flanking intron regions (20 bp) of 20099 genes in the human whole exome. Then, we compared the sequencing data with the human genome hg19 (GRCh37) reference sequence and evaluated the coverage and sequencing quality of the target area. We obtained 1523 genes related to the phenotype of the subject through multiple database searches.

The article "A novel TUBG1 mutation with neurodevelopmental disorder caused by malformations of cortical development" was retracted in 2023. Reasons: suspected computer-generated content; unreliable results or conclusions; concerns about the data; concerns about the results or conclusions.

This test analyzes the copy number variant sequencing (CNV-Seq) of large fragments (two or more consecutive exons) of the listed genes, and the CNVs have been verified by orthogonal experiments (qPCR or MLPA). When a detected pathogenic or possibly pathogenic variant is in an autosomal-recessive gene, the laboratory ensured that the coverage of the gene coding sequence reaches 100% through NGS and/or Sanger sequencing.

### 2.4. Analysis of Whole Exome Sequencing Data

First, we conducted mutation search and mutation annotation processes and found all possible mutations. Then, public databases (ESP6500, 1000 Genomes, ExAC, GnomAD) were used to exclude all mutations detected in the patient's sequencing data with a frequency greater than 0.001. By searching the OMIM, Swiss-Var, HGMD and ClinVar databases, we annotated reported disease genes and reported pathogenic sites. For missense mutations that are not recorded in the database, we used Polyphen-2, SIFT, CADD, and Mutationtaster protein software to predict the harmfulness of protein function. Finally, we combined the results of the WES and CNV-Seq analysis with the patient's phenotype, EEG and MRI analysis, and we performed genetic analysis according to the pathogenicity assessment results according to the ACMG guidelines.

According to the mutations found in WES, primers were designed, and Sanger sequencing was performed by polymerase chain reaction amplification to verify the mutation and inheritance pattern of WES.

## 3. Results

CNV-Seq detection did not find duplication or deletion of fragments. By WES, we analyzed the human GRCh37/hg19 genome database and found a heterozygous variant of *TUBG1* at chr17: 40765924 (NM_001070.4, *TUBG1*: c.751A>T; p.N251Y) adenine 751 was changed to thymine in the coding region and the aspartic acid encoding the protein became a tyrosine. The parent of the patients did not present the variant by WES, so the de novo variant was verified by Sanger sequencing (Figure 3(a)) and was not detected in the published database. The C.751A>T variant is not reported in HGMD or ClinVar databases or the published literature. Functional prediction indicated that the variant was more likely to cause changes in protein structure and function. Based on the patient's phenotype in conjunction with ACMG guidelines (PS2 + PM2 + PP3), this variant was evaluated as likely pathogenic.

The article "A novel TUBG1 mutation with neurodevelopmental disorder caused by malformations of cortical development" was retracted in 2023. Reasons: suspected computer-generated content; unreliable results or conclusions; concerns about the data; concerns about the results or conclusions.

Through analysis of protein conservation at *TUBG1:* c.751A>T; p.N251Y, the aspartic acid protein structure in this region of multiple species is highly conserved (Figure 3(b)).

We used Model V2.0 software to predict the complete structure of the *TUBG1* protein, and the visualization was produced using SAVES5.0. The three-dimensional structure diagram of wild-type and c.751A>T; p.N251Y *TUBG1* mutant protein reveals that the three-dimensional structure of the mutant protein was altered. This change may have a pathogenic effect on body function, leading to the occurrence of neurodevelopmental disorders caused by MCD (Figure 3(c)).

## 4. Discussion

Neurodevelopmental disorders caused by MCD are very rare neurological diseases. MCD represents a large group of brain cortical anomalies characterized by distinctive MRI findings [3]. The diagnosis of MCD is challenging due to frequent difficulties in defining etiologies. MRI is an essential diagnostic tool used in the assessment of specific epileptogenic cortical malformations or syndromes [14], but no specific cause could be detected. At present, thirteen cases of *TUBG1* mutations have been reported globally (Table 1). These cases cannot be diagnosed using chromosomal microarrays or biochemical screening for congenital metabolic abnormalities [15, 16]. In this study, we detected the etiology by whole-exome sequencing combined with CNV-Seq, but CNV-seq did not find duplications or deletions of fragment. We found that the *TUBG1* gene c.751A>T; p.N251Y is a novel pathogenic variant by WES, and the patient was finally diagnosed.

***γ***-Tubulin (*TUBG1*) was first described by Oakley and Oakley [17]. It belongs to the tubulin superfamily (including *TUBA1A*, *TUBB2A*, *TUBB2B*, *TUBB3*, *TUBB4A*, *TUBB*, and *TUBG1*). These tubulin gene mutations are related to a series of cortical malformations by disrupting normal microtubule interactions, which further affect the proliferation, migration, and differentiation of neuronal cells, as well as the growth and guidance of axons. Moreover, these genes are related to a series of brain malformations [18–20]. The *TUBG1* mutant affects the location of neurons and interferes with the movement of newborn neurons but does not affect the proliferation of progenitor cells [5]. The latest research suggests that novel heterozygous missense variants in the tubulin *TUBG1* gene lead to malformations of human cortical development, which further leads to intellectual disability and epilepsy [21].

The article "A novel TUBG1 mutation with neurodevelopmental disorder caused by malformations of cortical development" was retracted in 2023. Reasons: suspected computer-generated content; unreliable results or conclusions; concerns about the data; concerns about the results or conclusions.

Thirteen patients with different MRI features of MCD caused by mutation of *TUBG1* have been reported. Poirier et al. (2013) first reported the cases of three patients with unrelated cortical hypoplasia. Two patients showed severe malformation of the corpus callosum and cortical thickening and 1 patient presented a moderate malformation of the corpus callosum [2]. Brock et al. (2018) reported the cases of eight patients with cortical hypoplasia. One patient had diffuse anencephaly, and seven had corpus callosum malformations. Six of seven patients mainly had frontal lobe deformities, and 1 patient presented an enlarged frontal and parietooccipital lobe [1]. Yuen et al. (2019) reported one patient with corpus callosum malformation, and another with a decrease in the number of the cerebral sulci and gyri [22]. MRI analysis of this patient showed bilateral thickening of the cerebral hemispheres (parietal, occipital and temporal lobes). The cortex was thickened, and the surface was smooth. Only a few shallow sulci were noted, and the brain parenchyma was normal.

Although the novel *TUBG1* variant has not been assessed in animal function experiments to confirm the relationship between its phenotype and genotype of MCD, we used Model V2.0 software to predict the structural integrity of *TUBG1* c.751A>T; p.N251Y variant protein and compared with the wild-type protein structure of the variant. We analyzed the putative effects of variants on protein structure and function. The three-dimensional structure diagram of wild-type and c.751A>T; p.N251Y *TUBG1* mutant protein reveals that the three-dimensional structure of the mutant protein is altered. The p.N251Y mutation transforms the structure from an extended strand to random coil as confirmed by the secondary structure prediction of *TUBG1* using the online HNN program. Based on the protein structure and function software prediction of the novel variant, we hypothesize that changes in the variant structure may affect the corresponding functions to produce pathogenic effects and lead to neurodevelopmental disorders caused by MCD.

Although the complete phenotypic spectrum of tubular proteinosis is not completely clear, the MRI of the patient and the phenotype of left auricle deformity in this report increase the phenotypic characteristics of tubular protein lesions and also indicate the high clinical heterogeneity of neurodevelopmental disorders. Further functional studies will be focused on the relationship between this rare variant site and the phenotype to elucidate disease mechanisms that may facilitate the development of targeted treatments.

The article "A novel TUBG1 mutation with neurodevelopmental disorder caused by malformations of cortical development" was retracted in 2023. Reasons: suspected computer-generated content; unreliable results or conclusions; concerns about the data; concerns about the results or conclusions.

Retrospective analysis of the *TUBG1* variant reveals that is almost entirely a de novo mutation [1, 2, 22]. It is difficult to implement early screening, and this condition lacks effective treatment measures. Therefore, prenatal diagnosis during pregnancy is an effective means to block the continuation of the genetic factors implicated in the disease. At present, only symptomatic treatment is available. This patient mainly underwent antiepileptic drug treatment and rehabilitation training. No convulsions occured in the 1-year follow-up, and the condition did not develop.

## 5. Conclusions

This study clarifies the genetic etiology of the neurodevelopmental disorders in the patient and further reveals its characteristic phenotypic spectrum, molecular genetic findings, and functional consequences of novel pathogenic *TUBG1* variants in neurodevelopmental disorder caused by MCD. This study provides important guidance for research on the pathogenesis, treatment, prognostic evaluation, and reproductive implications of this disease.

## Figures and Tables

**Figure 1:** (a) The patient's family diagram. (b) The patient's facial features and images of both ears with left auricle deformity and a lack of an auricle structure.

**Figure 2:** Magnetic resonance imaging of the patient's brain. (a) Female patient aged 8 years and 9 months. Magnetic resonance imaging of the brain showed the gyrus of each lobe of the bilateral cerebral hemispheres is thick, the cortex is thickened, the surface is smooth, the sulci are few and shallow, and the bilateral ventricles are enlarged. The white arrow indicates the deformity of the corpus callosum; (b, c, d) Show the T1W1, T2W1, and T2W1 FLAIR signals of the parietal lobe, respectively; (e, f, g) show the T1W1, T2W1, and T2W1 FLAIR signals of the temporal lobe and occipital lobe, respectively.

**Figure 3:** Analysis of the *TUBG1*:c.751A>T; p.N251Y mutation. (a) Sanger sequencing of the child suggested a de novo mutation in the proband. (b) *TUBG1* gene c.751A>T p.N251Y protein conservation analysis diagram. (c) Three-dimensional structures of *TUBG1* (WT) and *TUBG1* (p.N251Y) protein. (A) Complete protein structure of TUBG1 predicted by ModellerV2.0 and visualized with SAVES5.0. (B) The structures of p.251N and p.251Y are presented as purple sticks. The p.N251Y mutation turn forms the structure from an extended strand to a random coil as confirmed by the secondary structure prediction of *TUBG1* using the online HNN program. This system encompasses a neural network algorithm for secondary structure prediction. The ‘h,' ‘e,' and ‘c' descriptors indicate the alpha helix, beta sheet, and random coil, respectively.

The article "A novel TUBG1 mutation with neurodevelopmental disorder caused by malformations of cortical development" was retracted in 2023. Reasons: suspected computer-generated content; unreliable results or conclusions; concerns about the data; concerns about the results or conclusions.

**Table 1:** Genotype and phenotype information of 13 previously reported *TUBG1* variants.

Case	Sex	Age at follow-up	Mutation	Mode of inheritance	Epileptic	Intellectual disability	Speech delay	Cortical dysgenesis (MRI)
This study	Female	8 years and 9 months	c.751A > T, p.Asn251Tyr	De novo	Yes	Severe	Can repeat words, cannot count or communicate	Bilateral thickening of the Guri of the lobes of the cerebral hemispheres, the cortex
Patient 1	Female	21 years	c.1160 T > C; p.Leu387Pro	De novo	Yes	Severe	Not available	Severe posterior predominant pachygyria/agyria (posterior agyria, frontal pachygyria), thickened cortex
Patient 2	Male	18 months	c.275A > G; p.Tyr92Cys	De novo	Yes	Severe	Not available	Severe posterior predominant pachygyria/agyria (posterior agyria, frontal pachygyria), thickened cortex
Patient 3	Female	31 years	c.991A > C; p.Thr331Pro	Father's DNA not available	Yes	Moderate	Not available	Posterior pachygyria, moderate posterior subcortical band heterotopia
Patient 4	Male	33 years	c.63C > A; p.Phe21Leu	De novo	No	Severe	Only sounds, no speech	Posterior predominant pachygyria (posterior frontal lobe and parieto-occipital cortex)
Patient 5	Male	21 years	c.985G > T; p.Asp329Tyr	Father's DNA not available	Yes	Severe	Nonverbal	Diffuse agyria
Patient 6	Female	19 months	c.776C > T; p.Ser259Leu	De novo	Yes	Not available	Delayed	Posterior predominant pachygyria (mild over frontal lobes, moderate over posterior lobes), cortex 10-13 mm thick
Patient 7	Female	14 years	c.776C > T; p.Ser259Leu	De novo	Yes	Not available	Nonverbal	Posterior predominant pachygyria, sparse cells over occipital lobes, cortex 13-15 mm thick
Patient 8	Female	11 years and 6 months	c.776C > T; p.Ser259Leu	Germline mosaicism in parent	Yes	Moderate	50 words	Posterior predominant pachygyria (mild over frontal lobe, moderate over temporal and occipital lobes), cortex 6-13 mm thick
Patient 9	Male	9 years and 6 months	c.776C > T; p.Ser259Leu	Germline mosaicism in parent	Yes	Moderate	Nonverbal	Posterior predominant pachygyria (mild over frontal lobe, moderate over temporal and occipital lobes), cortex >15 mm thick
Patient 10	Male	15 years	c.769A > T; p.Ile257Phe	De novo	Yes	Moderate	5 word sentences	Posterior predominant pachygyria (almost normal over frontal lobes, pachygyria over perisylvian and occipital lobes), cortex 6-10 mm thick
Patient 11	Female	18 months	c.776C > T; p.Ser259Leu	De novo	Yes	Severe	Nonverbal	Posterior predominant pachygyria (mild over frontal lobe, moderate over temporal and occipital lobe, deep parietal lobe infolding)
Patient 12	Female	10 years	c.202G > A; p.Asp68Asn	De novo	No	Moderate	Normal	Posterior predominant pachygyria, band heterotopia, nodular heterotopia
Patient 13	Male	6 months	c1021C > T; p.Arg341Trp	De novo	Yes	Moderate global delay	Moderate global delay	Reduced cortical sulci and gyri

The article "A novel TUBG1 mutation with neurodevelopmental disorder caused by malformations of cortical development" was retracted in 2023. Reasons: suspected computer-generated content; unreliable results or conclusions; concerns about the data; concerns about the results or conclusions.

## Data Availability

The data used to support the findings of this study are all included within the article.
